# Intense intestinal carriage and subsequent acquisition of multidrug-resistant enterobacteria in neonatal intensive care unit in Morocco

**DOI:** 10.1371/journal.pone.0251810

**Published:** 2021-06-30

**Authors:** Btissam Arhoune, Samira El Fakir, Sara Himri, Kaoutar Moutaouakkil, Salma El Hassouni, Moussa Benboubker, Fouzia Hmami, Bouchra Oumokhtar

**Affiliations:** 1 Laboratory of Microbiology and Molecular biology, Faculty of Medicine and Pharmacy, Sidi Mohammed Ben Abdellah University, Fez, Morocco; 2 Laboratory of Epidemiology and Clinical Research, Faculty of Medicine and Pharmacy, Sidi Mohammed Ben Abdellah University, Fez, Morocco; 3 Neonatal Intensive Care Unit, University Hospital Hassan II, Fez, Morocco; University of Nicolaus Copernicus in Torun, POLAND

## Abstract

This study was conducted in order to know the colonization rate of MDR enterobacteria in neonates during their hospitalization in neonatal intensive care unit (NICU). Furthermore, we investigated risk factors for potential colonization and molecular epidemiology of isolated resistant bacteria. This prospective study was carried out in the neonatology and intensive care unit department of the University Hospital of Fez (Morocco) from February 2013 to July 2015. All consecutive admitted newborns were screened for intestinal and nasal carriage of MDR enterobacteria at admission of the babies and during the hospitalization. During the study period, a total of 641 *Enterobacteriaceae* were isolated and *Klebsiella pneumoniae* was the predominated bacteria. Bacterial identification and antibiograms were performed according to the international standards. On admission, 455 newborns were screened. A median age of these newborns was 1 day with an extended 147 days and their average weight was 2612 ± 1023 grams. 22.4% of neonates were found colonized by an ESBL producing *Enterobacteriaceae* (ESBL-E), 8.7% by a carbapenemases producing *Enterobacteriaceae* (CPE). During hospitalization, 207 of newborns were included in the acquisition study. 59.4% of newborns acquired an ESBL-E during their stay, 12.5% has acquired CPE. The *bla*_*CTXM-15*_ gene was the most frequently detected (81.2%) among ESBL-E. While, all CPE has expressed the *bla*_*OXA-48*_ gene exclusively. Two risk factors have been significantly associated with MDR enterobacteria colonization at admission which are newborns admission from maternity of the university hospital (95% CI, 1.859–5.129, P = 0.000) and neurological distress (95% CI, 1.038 to 4.694, P = 0.040). During hospitalization, the none risk factor was significantly associated with the carriage of MDR-E. The high rate of colonization, the MDR enterobacteria and the resistance genes found represent good indicator of cross-transmission in the NICU. An active strategy to control the spread of MDR enterobacteria should be applied.

## Introduction

Multidrug-resistant *Enterobacteriaceae* (MDR-E) occurring in health care settings cause several healthcare associated infections (HAI), particularly bacteremia (45%), pneumonia (22%), gastrointestinal infection (8%), and urinary tract infection (5%) [1]. These infections remain a major cause of mortality and morbidity among hospitalized newborns, especially premature infants and babies with low birth weight [2–4]. According to the World Health Organization, HAI account from 4 to 56% of all causes of neonatal death among infants hospitalized in developing countries. It can attain 75% in Southeast Asia and Africa [5].

Newborns admitted to the neonatal intensive care unit (NICU) are frequently colonized by MDR bacteria. The risk factors related to this colonization has been widely reported and can start from anamnestic factors through to risk factors related to invasive procedures associated with health care. The acquisition of MDR-E in the NICU may result from the increasing use of antibiotics or transmission from one patient to another due to caregivers and the hospital environment [6]. Neonatal sepsis caused by multidrug-resistant gram-negative organisms, particularly *Enterobacteriaceae* is a concern in premature infants, and treatment options are limited [7]. In low- and middle-income countries (LMICs), these infections are associated with poor outcomes and high mortality rates [8].

Outbreaks occurring in NICUs are often caused by *Enterobacteriaceae* producing Extended-spectrum beta-lactamases (ESBLs) or carbapenemases (CPEs). This is a particular concern because these resistances are encoding by genes carried on mobile genetic elements, facilitating patient-to-patient transmission. Furthermore, these genes may carry resistance to other antimicrobial classes, which amplifies the risk of therapeutic failure [9]. Most previous reports regarding the molecular characterization of ESBLs concluded that the CTX-M variant encoding the ESBL were predominating worldwide. While, the prevalence of carbapenemases variants reported such as KPC, IMP, and VIM varies depending on the areas of the region. The OXA-48 remains the cabapenemases most identified in Mediterranean countries.

Although early screening of newborns colonized with ESBL or carbapenemase-producing bacteria can potentially contribute to the prevention and control of late-onset infections, few studies are addressing this issue in hospital children [10]. We established a systematic screening of newborn at admission to studied the acquisition of multidrug resistant bacteria. We reported, in previous work, the acquisition rate of *Acinetobacter baumannii* through hospitalized newborns. In the present study, we address the problem of MDR *Enterobacteriaceae* involved during newborn hospitalization. It aims to describe the colonization rate, risk factors and the molecular epidemiology of the bacteria involved during hospitalization.

## Methods

### Study

This prospective study was conducted at the neonatology and intensive care unit department of a University Hospital of Fez (Morocco) from February 2013 to July 2015. The setting was a medical and surgical NICU which has 18 beds divided into 2 sectors (9 beds were in each one); sector 1 corresponds to an intensive care unit and sector 2 corresponds to a pretermbaby unit. This NICU is the only one in Fez city (center of Morocco) with a population estimated approximately at 1.5 million inhabitants. Three seniors, 8 physicians, and 6 nursesare assigned to this ward daily.

### Patients

During this period, all consecutive neonates admitted into the unit are included. Only the first NICU admission per neonate was included in the analysis. Neonates hospitalized during the week end, which have died or output before 48h of hospitalization were excluded. Babies were evaluated for *Enterobacteriaceae* intestinal (a) carriage at admission and (b) acquisition during hospitalization. Imported carriers and those without follow-up samples (due to death or discharge before the scheduled follow-up sampling) were excluded from acquisition analysis.

### Ethics committee

Ethical approval was obtained from the local ethics committee in the University Hospital Center Hassan II in Fez- Morocco and all the parents’ babies were informed of the conditions related to the study and gave their written, informed consent.

### Statistical analysis

Potential risk factors associated with *Enterobacteriaceae* colonization were studied. The sociodemographic and clinical characteristics of patients were collected prospectively by using a standard written questionnaire. The statistical analysis for our study was done using SPSS, version 20 (SPSS Inc., Chicago, IL, USA) software. It consisted primarily to describe the study population. Results for quantitative variables were presented as mean ± standard deviation and for qualitative variables; results were presented as number (percentage). Then, a univariate analysis was performed to establish all associations between gender, age, birth weight, prematurity, birthplace, admission route, delivery mode, date of hospital and NICU admission, and diagnosis on NICU admission. Antimicrobial therapy, breastfeeding, central or peripheral venous catheterization, and length of hospital stay were also recorded in the questionnaire. Chi-square test and fisher’s exact test were used to establish significant association as appropriate. The *P* < 0.05 was deemed statistically significant. The multivariate analysis was performed to identify potential risk factors associated with intestinal *Enterobacteriaceae* multi-drug-resistant colonization using simple logistic regression analysis. All variables with p < 0.2 in univariate analysis were included in a logistic regression model for multivariate analysis. Odds ratios were presented with the corresponding 95% confidence intervals (OR, CI 95%).

### Sampling and screening

Two rectal swabs were collected from each newborn. The initial sample was performed up to 6 hours from admission to the NICUs and the second one after 5 days of hospitalization. Rectal swab specimens were enriched in nutrient broth BHI (Brain Heart infusion, Oxoid®) at 37°C for 24h. Then, they were inoculated on Mac Conkey agar plates and then incubated at 37° C for 24h. The identification of *Enterobacteriaceae* isolates was performed by classical bacteriological techniques and confirmed by using API20E galleries (Biomérieux, Marcy l’Etoile, France).

### Antimicrobial susceptibility testing

Antimicrobial susceptibility was determined as recommended by the EUCAST 2013, the following antimicrobial agents (Oxoid®) were tested: amoxicillin (10 mg); amoxicillin/clavulanic acid (20/10mg); cefalotin (30mg); cefotaxime (30mg); céftazidime (30mg); ertapenem (10 mg); nalidixic acid (30 mg); ciprofloxacin (5 mg); norfloxacin (10 mg); gentamicin (10 mg); amikacin (30mg); fosfomycin(50mg); and trimethoprim/sulfamethoxazole (SXT) (1.25/23.75 mg). *Enterobacteriaceae* isolates resistant to three or more classes of antibiotics were considered as MDR. ESBL production was screened by the double-disk synergy test. The standard strains *E*. *coli* ATCC 25922 were used as negative control strains for ESBL production. The modified Hodge test was performed for screening carbapenemases production to all ertapenem resistant isolates.

### Preparation of DNA template for PCR

Total DNA was extracted by suspending a few colonies of an overnight culture of *Enterobacteriaceae* isolates in 500μL of DNase- and RNase-free water (Invitrogen, Paisley, UK). The suspension was boiled at 100°C for 10min in a thermal block (Polystat 5, Bioblock Scientific, France), then centrifuged at 14000 x *g* for 10 min. An aliquot of 2 μL of the supernatant was used as a DNA template for PCR.

### Detection of β-lactamase- and carbapenemase-encoding genes

All DNA from ESBLE and CPE isolates have been stored at -20°C for detection of subsequent resistance genes. Therefore, All ESBL-producing strains were screened by PCR as described previously for the following β-lactamase-encoding genes: *bla*_*CTX-M*_ phylogenetic lineage groups 1, 2, and 9; *bla*_*TEM*_; and *bla*_*SHV*_. The *bla*_*OXA-48*_,*bla*_*KPC*_,*bla*_*NDM*_, *bla*_*IMP*,_ and *bla*_*VIM*_ genes were also detected to confirm the presence of carbapenemase-encoding genes. The known β-lactamase-producing strains, recuperated from Pasteur institute of Morocco, *E*. *coli* U2A1790(CTX-M-1), *E*. *coli* U2A1799 (CTX-M-9), *Salmonellasp*. U2A2145(CTX-M-2), *Salmonella sp*. U2A1446 (TEM-1 and SHV-12) were used as positive controls. The known carbapenemase-producing strains were used as positive controls. PCR products were detected on 1.5% agarose gels (FMC BioProducts, Rockland, ME) following ethidium bromide staining and ultraviolet illumination, and were photographed with an Olympus digitalcamera (Olympus Soft Imaging Solutions GmbH, Münster, Germany).

### Sequencing of resistance genes

All amplified products obtained were sequenced to validate their identities. Both strands of the purified amplicons were sequenced with the same primers used for PCR amplification. The nucleotide and deduced protein sequences were analysed with software available on the Internet at the National Center for Biotechnology Information (NCBI) website (http://www.ncbi.nlm.nih.gov).

## Results

### Study population

During the study period, 455 neonates met the criteria for inclusion were swabbed at admission to the NICU. The average gestational age and mean birth weight were 35.2 (±3.2) weeks and 2612.1 g (±1023.2) respectively. 150 were carriers of MDR *Enterobacteriaceae* at admission. Of the 305 non-carriers, just 207 had follow-up rectal swabs discharge. The remaining 98 patients were excluded from acquisition analysis because they were discharged or died before the scheduled sampling (Fig 1).

**Fig 1:** Flowchart of the patients.

### MDR *Enterobacteriaceae* intestinal carriage

During the study period, a total of 641 *Enterobacteriaceae* were isolated. *Klebsiella pneumoniae* was the predominated bacteria (n = 319), followed by *Escherichia coli* (n = 261). Furthermore, 17 strains of *Enterobacter cloacae*, 16 of *Klebsiella oxytoca*, 10 of *Citrobacter freundii*, 9 of *Proteus mirabilis*, 4 of *Morganella morganii*, 1 of *Enterobacter aerogenes*,1 of *Proteus vulgaris*, 1 of *Citrobacter braakii*, 1 of *Providencia stuartii*, and1 of *Serratia marcescens* were isolated.

In the current work, 33% of admitted newborns were carriers of MDR *Enterobacteriaceae* (150/455). We noted that 22.4% of all strains were producers of ESBL resistance and 8.7% were producers of carbapenemases resistance. Usually, MDR *E*. *coli* species was the most identified in this carriage (50.6%).

During NICU stay, the prevalence of MDR *Enterobacteriaceae* intestinal acquisition was 64.2% and 92.4% of them were ESBL producers. This time, MDR *K*. *pneumoniae* was the most predominant species acquired (88.7%). The prevalence of the different resistance types found in *Enterobacteriaceae* (ESBL and carbapenemases) were shown in Table 1.

**Table 1:** Prevalence of ESBL and CARBA carriage among newborns hospitalised in NICU.

*Enterobacteriaceae*	Carriers at admission* N = 455[%(N)]	Colonised during NICU stay* N = 207[%(N)]
**MDR-*Enterobacteriaceae***	**33 (150/455)**	**64.2 (133/207)**
ESBL**-*Enterobacteriaceae***	22.4 (102/455)	59.4 (123/207)
ESBL**-***K*. *pneumoniae*	77.4 (79/102)	94.3 (116/123)
ESBL**-***E*.*coli*	32.3 (33/102)	26 (32/123)
ESBL**-**Other species	8.8 (9/102)	8.1 (10/123)
CARBA**-*Enterobacteriaceae***	8.7 (40)	12.5 (26/207)
CARBA*-K*. *pneumoniae*	42.5 (17/40)	46.1 (12/26)
CARBA*-E*.*coli*	45 (18/40)	61.5 (16/26)
CARBA**-**Other species	12.5 (5/40)	7.6 (2/26)

*Carriage of at least one MDR *Enterobacteriaceae* isolate.

### Risk factors of MDR *Enterobacteriaceae* carriage

Univariate analysis performed between patient characteristics and intestinal carriage of MDR-*Enterobacteriaceae* on admission had shown that 57.3% of admitted newborns aged younger than 48h were carriers of MDR-E (p = 0.001). In addition, 54.7% of non-breastfed babies were found colonized at admission (p = 0.042) (Table 2).

**Table 2:** Association between patient’s characteristics and prevalence of multidrug-resistant *Enterobacteriaceae* carriage on the day of admission and during hospitalization at NICU.

		At admission				During NICU stay			
Category		Patients numbers (%)	MDR-EB -	MDR-EB +*	p-value	Patients numbers (%)	MDR-EB -	MDR-EB +	p-value
		n = 455	[N (%)]	[N (%)]		n = 207	[N (%)]	[N (%)]	
**Gender**	Male	267 (58.7)	180 (59)	87 (58)	0.457	124 (59.9)	36 (65.5)	88 (57.9)	0.207
	Female	188 (41.3)	125 (41)	63 (42)		83 (40.1)	19 (34.5)	64 (42.1)	
**Age (days)**	0–2	Mean±SD	222 (72.8)	86 (57.3)	**0.001**	Mean±SD	39 (70.9)	112 (73.7)	0.408
	> 2	6.5±15.8	83 (27.2)	64 (42.7)		5.1±12.2	16 (29.1)	40 (26.3)	
**Prematurity**	Yes	224 (49.2)	156 (51.1)	68 (45.3)	0.140	113 (54.6)	29 (52.7)	84 (55.3)	0.433
	No	231 (50.8)	149 (48.9)	82 (54.7)		94 (45.4)	26 (47.3)	68 (44.7)	
**Birth weight (g)**	< 2500	Mean±SD	158 (51.8)	68 (45.3)	0.115	Mean±SD	31 (56.4)	81 (53.3)	0.408
	≥ 2500	2612±1026g	147 (48.2)	82 (54.7)		2466±975	24 (43.6)	71 (46.7)	
Pathology**	Respiratory distress	259 (56.9)	182 (59.7)	77 (51.3)	**0.056**	123 (59.4)	32 (58.2)	91 (59.9)	0.475
	Icterus	38 (8.4)	21 (6.9)	17 (11.3)	0.078	14 (6.8)	2 (3.6)	12 (7.9)	0.229
	Surgical pathology	31 (6.8)	17 (5.6)	14 (9.3)	0.099	11 (5.3)	4 (7.3)	7 (4.6)	0.328
	Neonatal suffering	34 (7.5)	24 (7.9)	10 (6.7)	0.401	16 (7.7)	4 (7.3)	12 (7.9)	0.573
	Neonatal infections	35 (7.7)	20 (6.6)	15 (10)	0.134	16 (7.7)	3 (5.5)	13 (8.6)	0.342
	Neurological distress	44 (9.7)	34 (11.1)	10 (6.7)	0.086	22 (10.6)	3 (5.5)	19 (12.5)	0.112
	Congenital malformations	11 (2.4)	9 (3)	2 (1.3)	0.239	6 (2.9)	2 (3.6)	4 (2.6)	0.505
	Others	49 (10.8)	29 (9.5)	20 (13.3)	0.141	18 (8.7)	7 (12.7)	11 (7.2)	0.168
**Birthplace**	Maternity of UH Fez	265 (58.2)	190 (41.8)	75 (50)	**0.026**	125 (60.4)	33 (60)	92 (60.5)	0.703
	Other hospital	164 (36)	97 (31.8)	67 (44.7)		66 (31.9)	19 (34.5)	47 (30.9)	
	Home	26 (5.7)	18 (5.9)	8 (5.3)		16 (7.7)	3 (5.5)	13 (8.6)	
**Admission route**	Maternity of UH Fez	235 (51.6)	178 (58.4)	57 (38)	**0.000**	117 (56.5)	31 (56.4)	86 (56.6)	0.870
	Other hospital	124 (27.3)	77 (25.2)	47 (31.3)		56 (27.1)	16 (29.1)	40 (26.3)	
	Home	96 (21.1)	50 (16.4)	46 (30.7)		34 (16.4)	8 (14.5)	26 (17.1)	
**Delivery mode**	vaginal	310 (68.1)	205 (67.2)	105 (70)	0.312	142 (68.6)	34 (61.8)	108 (71.1)	0.137
	Caesarean section	145 (31.9)	100 (32.8)	45 (30)		65 (31.4)	21 (38.2)	44 (28.9)	
**Venous Catheterization**	peripheral	--	--	--	--	203 (98.1)	55 (100)	148 (97.4)	0.288
	central	--	--	--		4 (1.9)	0 (0)	4 (2.6)	
**Breastfeeding**	Breastfed newborn	179 (39.3)	111 (36.4)	68 (45.3)	**0.042**	69 (33.3)	17 (30.9)	52 (34.2)	0.394
	Diet newborn	276 (60.7)	194 (63.6)	82 (54.7)		138 (66.7)	38 (69.1)	100 (65.8)	
**Antibiotherapy**	Ceftriaxone+gentamicin	--	--	--	--	116 (56)	35 (63.6)	81 (53.3)	0.121
	Aximicin+gentamicin	--	--	--		74 (35.7)	18 (32.7)	56 (36.8)	0.354

*Carriage of at least one MDR *Enterobacteriaceae* isolate

**Neonates may have more than one reason for hospitalization.

The same analysis was performed between patients’ characteristics and this time with the intestinal acquisition of MDR-E during hospitalization revealed that there is a significant association between the age < 48h (p = 0.001) and the acquisition of MDR-E during the stay. Any hospital stay ≥3 days (p = 0.007) was also linked to the acquisition of MDR-E. In other words, the results showed that 73.3% of newborns were younger than 48h at the time of admission and 96% of all babies which stayed at least 3 days in the ward were acquired an MDR-E (Table 2).

### Multivariate analysis

On admission, the multivariate analysis showed that newborns imported from maternity of university hospital (95% CI, 1.859–5.129, P = 0.000) were 3 times more likely to be carriers of MDR-E than those imported from their houses. Also, neonates with neurological distress are 2 times more likely to be carriers of MDR-E (95% CI, 1.038 to 4.694, P = 0.040) than those who do not have this pathology. Table 3 shows all the risk factors for the carriage of MDR-E defined in this study.

**Table 3:** Multivariable analysis for MDR-*Enterobacteriaceae* carriage at NICU admission and acquisition during hospitalization.

Variable	Multivariable analysis for MDR *Enterobacteriaceae* carriage at NICU admission	
	OR (95%CI)	P value
**Neurological distress**	2.207 (1.038–4.694)	0.040
**Imported from the maternity ward of the university hospital**	3.088 (1.859–5.129)	0.000
**Imported from other wards or institutions**	2.010 (1.251–3.230)	0.004

During hospitalization, the none risk factor was significantly associated with the carriage of MDR-E (Table 3).

### Antibiotic resistance

On admission, the study of the resistance profiles of *Enterobacteriaceae* concerning the different antibiotics tested among newborns showed a high resistance rate for Ampicillin (75.3%) followed by Amoxicillin associated with Clavulanic acid (53.9%). Ceftazidime or cefotaxime resistance was also high with 47.6%. However, the resistance rate to Amikacin was very low (0.9%).

During the hospital stay, the study of resistance patterns of *Enterobacteriaceae* isolated showed that almost all isolates are resistant to ampicillin (97%) and amoxicillin/clavulanic acid (92%). The rate of resistance to ceftazidime/cefotaxime was 89.9% and gentamicin was 82.9%. Half of the isolates were resistant to nalidixic acid and ciprofloxacin. While only 3% of the isolates were resistant to amikacin. The different resistance profiles found according to the bacterial species identified are presented in Table 4.

**Table 4:** Resistance profiles of the different *Enterobacteriaceae* isolated on admission and during hospitalization.

*Enterobacteriaceae* species (No.; %) n = 313	No. (%) of resistant isolates at admission									
	AMX	AMC	FOX	CTX/CAZ	GN	AK	NA	NOR/CIP	SXT	ETP
*E*. *coli* (n = 152; 48)	88	65	36	56	51	2	53	46	38	18
*K*. *pneumoniae* (n = 124; 39.6)	124	80	3	79	72	0	39	39	49	17
*E*. *cloacae* (n = 11; 3.5)	*	*	*	9	7	0	7	5	6	4
*K*. *oxytoca* (n = 10; 3.1)	1	1	0	1	1	0	1	1	1	1
*C*. *freundii* (n = 5; 1.5)	*	*	*	3	2	1	2	2	1	0
*P*. *mirabilis* (n = 5; 1.5)	1	1	1	1	0	0	0	0	0	0
*M*. *morganii* (n = 2; 0.6)	*	*	*	0	0	0	0	0	0	0
*C*. *braakii* (n = 1; 0.3)	1	1	1	0	0	0	0	0	0	0
*P*. *vulgaris* (n = 1; 0.3)	*	1	1	0	0	0	0	0	0	0
*P*. *stuartii* (n = 1; 0.3)	*	*	*	0	0	0	0	0	0	0
*S*. *marcescens* (n = 1; 0.3)	*	*	*	0	0	0	0	0	0	0
*Enterobacteriaceae* species (No.; %) n = 313	236 (75.3)	169 (53.9)	62 (19.8)	149 (47.6)	133 (42.4)	3 (0.9)	102 (32.5)	93 (29.7)	95 (30.3)	40 (12.7)
	**No. (%) of resistant isolates during NICU stay**									
	**AMX**	**AMC**	**FOX**	**CTX/ CAZ**	**GN**	**AK**	**NA**	**NOR/CIP**	**SXT**	**ETP**
*K*. *pneumoniae* (n = 195; 59.4)	195	184	10	184	169	0	95	90	99	18
*E*. *coli* (n = 109; 33.2)	100	96	63	93	89	9	79	77	28	26
*E*. *cloacae* (n = 6; 1.8)	*	*	*	6	3	1	3	3	3	2
*K*. *oxytoca* (n = 6; 1.8)	*	5	1	5	5	0	2	2	3	2
*C*. *freundii* (n = 5; 1.5)	*	*	*	4	3	0	1	1	0	1
*p*. *mirabilis* (n = 4; 1.2)	4	3	0	2	2	0	2	0	0	0
*M*. *morganii* (n = 2; 0.6)	*	*	*	1	1	0	0	0	0	0
*E*. *aerogenes* (n = 1; 0.3)	*	*	*	0	0	0	0	0	0	0
*Enterobacteriaceae* species (No.; %) n = 328	319 (97.2)	302 (92)	88 (26.8)	295 (89.9)	272 (82.9)	10 (3)	182 (55.4)	173 (52.7)	133 (40.5)	49 (14.9)

*Natural resistance

AMP: ampicillin; AMC: amoxicillin / clavulanic acid; FOX: cefoxitin; CTX: cefotaxim; CAZ: ceftazidim; GN: gentamicin; AK: amikacin; NA: nalidixic acid; NOR: norfloxacin; CIP: ciprofloxacin, SXT: cotrimoxazol; ETP: ertapenem.

### Molecular analysis

All isolates found resistant to C3G and/or imipenem were tested for resistance genes. Phenotypic tests confirming the production of ESBL or CARBA enzymes have been carried out including the synergy test and the Hodge test.

#### *Enterobacteriaceae* producing ESBL

Of the 641enterobacterial isolates collected during this study, 330 were confirmed as ESBL producers by the synergy test (51.4%). *K*. *pneumoniae* was the predominant specie with a frequency of 76.9% (254/330), while 16.6% of the isolates were *E*. *coli* (55/330).

The *bla*_*CTX-M-1*_ gene was the most dominant with a frequency of 81.2% (268/330), followed by *bla*_*SHV*_ with 69.6% (230/330). The *bla*_*TEM*_ was present in 44.2% of isolates and the *bla*_*CTX-M-9*_ in 20.4% of isolates. However, *bla*_*CTX-M-2*_ was detected only in 5.7% of strains. Sequence analysis confirmed the presence of the five nucleotide sequences *bla*_*CTX-M-1*,_ *bla*_*CTX-M-2*,_ *bla*_*CTX-M-9*,_ *bla*_*SHV*,_ *bla*_*TEM*_.

#### *Enterobacteriaceae* producing carbapenemases

The results of the antibiograms showed that 89 isolates are resistant to Imipenem and / or Ertapenem. *E*. *coli*.comes first with 44 isolates followed by *K*. *pneumoniae* with 35 strains. The Hodge test was used to select 42 positive isolates, which corresponds to 47%.

All Hodge positive isolates were screened for PCR production of carbapenemases. The results of the *bla*_*KPC*_, *bla*_*NDM*_, *bla*_*IMP*_, *bla*_*VIM*,_ and *bla*_*OXA-48*_ genes showed that all isolates *k*. *pneumoniae*, *k*. *oxytoca* and *E*. *coli* exclusively carried the *bla*_*OXA-48*_ gene. In contrast, isolates of *E*. *cloacae* and *C*. *freundii* did not harbor any of these genes. Sequence analysis confirmed the presence of the nucleotide sequence *bla*_*OXA-48*_.

## Discussion

The study of colonization by MDR *Enterobacteriaceae* in hospitalized newborns showed a high prevalence of these bacteria, whether on admission (33%) or during hospitalization (59%). Several risk factors make acquisition almost inevitable (from postpartum to hospitalization risk factors) but the high rate only suggests that the application of universal and additional precautions is not optimal in-hospital services especially with regard to small children whose infectious state is bacteriologically documented., it can contribute to a cross-transmission given the charge of work and the invasive multitude acts in the unit.

Several studies have evaluated the prevalence of ESBL-E colonization among patients hospitalized in ICUs [11].

The predominant resistance mechanism in our study is the production of ESBL; we reported an acquisition rate of 59%, which means that 59% of the patients became colonized with ESBL during their hospital stay. Detsis et al. reported that the risk of subsequent ESBL-E infection in colonized patients is approximately 50 times higher than in non-colonized patients, and thus ESBL-E colonization of the gastrointestinal tract may be a useful tool for predicting ESBL-E infection [12]. Also, these colonized newborns can serve as reservoirs for other newborns as well as for potential epidemics [13, 14].

Of the ESBL-producing enterobacteria, *K*. *pneumoniae* has been widely implicated in numerous nosocomial and neonatal epidemics worldwide [15]. This specie has been responsible for 16–28% of bacteremia cases in different parts of the world [16]. In this study, 94% of the ESBL acquisition cases consisted of acquisition of ESBL-producing *K*. *pneumoniae*, which is consistent with another Italian report [17].

Also, the most recent challenge has been the spread of carbapenemase-producing *Enterobacteriaceae* (CPE) around the world [12]. We found that 8.7% of screened patients were colonized with CPE on admission and 12.5% during their stay. A recent study reported a CPE rate of 1.6% among newborns hospitalized in Algeria. This resistance was encoded exclusively by the *bla*_*OXA-48*_ gene [13].

Frequently colonizing of admitted newborns are *K*. *pneumoniae* and *E*. *coli*, which are common enterobacteria in the intestinal tract of hospitalized newborns. Both bacteria are naturally susceptible to many antibiotics but can develop resistance to many drugs, particularly beta-lactam antibiotics, the most commonly used antibiotics in NICUs. This resistance is a consequence of the selection pressure due to the excessive use of antibiotics and of their strong genetic determinism that gives them a high power of diffusion [19].

A high frequency of resistance to commonly used antibiotics such as cephalosporin 3G or gentamicin was observed in the isolates identified during our study. We noted that 90% of ESBL-E and 95% of EPCs, were resistant to gentamicin as well. More than 80% of these bacteria have co-resistance with quinolones and fluoroquinolones. Moreover, several authors have observed the same broad spectrum of resistance in enterobacterial strains isolated from hospitalized infants [14–16].

In recent decades, the predominant genotype in β-lactamase-producing enterobacteria has shifted from TEM and / or SHV to CTX-M (genes encoding ESBL). The prevalence of these genes varies widely. In Saudi Arabia, rates of 97.3% for SHV and 84.1% for TEM have been reported [17]. In contrast, in France, Birgy et al. reported lower rate: 6.3% and 9.4% respectively for TEM and SHV [18]. For the CTX-M β-lactamase, the *bla*_*CTX-M-1*_ group was the most detected in our work. An earlier study carried out in Morocco on isolates of ESBL-producing *E*. *coli* showed agreement (80%) with our results [19]. In South Asia, the CTX-M-1 and CTX-M-9 groups were identified, but none CTX-M-2 [17]. However, CTX-M-2 is more prevalent in most South American countries [20].

Subgroup *bla*_*CTX-M-1*5_ is considered the most common type of ESBL worldwide [21–23]. In Moroccan hospitals, CTX-M-15 and CTX-M-28 were the two CTX-M enzymes identified in patients [19]. In the present study, *bla*_*CTX-M-15*_ was the only subclass found among all isolates harboring the *bla*_*CTX-M-1*_ gene.

On the other hand, the enzyme OXA-48 is a group D of β-lactamase, having the greatest catalytic property to imipenem, it also hydrolyzes penicillins and spares wide-spectrum cephalosporins. This enzyme, encoded by the *bla*_*OXA-48*_ gene, was initially identified from a strain of *K*. *pneumoniae* isolated in Turkey [24]. This gene is localized on a plasmid and has also been identified in *E*. *coli* and *Citrobacter freundii*, but not in *A*. *baumannii* [25]. Moreover, this corresponds to the results published in our previous manuscript which shows that all isolates of *A*. *baumannii* harbored *bla*_*OXA-23*_ and *bla*_*OXA-51*_ but no *bla*_*OXA-48*_ [26].

The identification of risk factors favoring the colonization of hospitalized newborns by MDR-E allows putting in place preventive strategies of transmission of MDR-E in health care structures. In SNRNs, the most commonly reported factors are birth weight; gestational age, use of invasive devices, previous treatment with antibiotics, and length of stay [27, 28].

The length of hospital stay as a risk factor has been associated with the acquisition of ESBL-E in neonates [29] as well as in adults hospitalized in ICUs [30]. On the other hand, inappropriate antibiotic therapy associated with ESBL-E colonization may result in prolonged hospital stays. Thus, the longer the hospital stay, the greater the risk of the onset of nosocomial bacteremia [31].

We also found that neurological distress and the origin from another hospital service presents risk factors associated with the carriage of an MDR-E on admission. Indeed, 38% of newborns coming from the maternity hospital of Fez University Hospital are carriers of MDR-E. These patients then constitute an important reservoir of MDR-E and will contribute, often through the hands of the medical staff, to the transmission of these bacteria to other hospitalized newborns. In the same context, Khiev and Veber reported that an intra- or extra-institutional transfer for hospitalization increases the risk of MDR-E colonization [32].

Cross-transmission of MDR-E between newborns through the environment and health care personnel remains the most likely route of newborn colonization. The prevention of colonization by MDR-E among hospitalized infants remains difficult. However, admission screening allows early detection of colonized patients and helps control the spread of these strains through the application of several appropriate control measures [33, 34].

The NICU of University Hospital Hassan II provides services to more than 1200 patients a year and drains a very important population that it is from the region of Fez than elsewhere. Building additional NICUs capacity in the region would help reduce local load and demand, thereby reducing the risk of transmission and infection.

Such as in many developing countries, low observance of hand hygiene practices among health professionals has been noted. Moreover, this situation amplifies the risk of transmission and spread of epidemic strains.

Any strategy for preventing MDR-E transmission and nosocomial infection is based primarily on respect for hand hygiene. Staff training is therefore an important element to succeed in this challenge.

In this context, we have developed and implemented a multimodal strategy focused on two different programs, the first is based on the implementation of hand hygiene and the optimization of standard and universal precautions. The second program is oriented towards the management of patients on the unit, starting with the systematic screening of newborns following childbirth at the hospital institutions and a reporting system for patients who have an infectious status that requires the initiation of the isolation or the cohorting of cases.

Our study has some limitations to consider. First, the moment of discharge screening can lead to biased estimates of the association between length of stay and MDR-E acquisition. Second, we did not evaluate for non-β-lactamase mechanisms of resistance such as those that relate to reduced outer membrane permeability, as we preferred to focus on resistance mechanisms with a high predilection for patient-to-patient transmission. Third, we were unable to carry out molecular analyses earlier, which led us to delay the publication of our results. at the same time, the inventory conducted very recently (in 2020) of the neonatal unit showed that the frequency of colonization is still high (around 60%). Last, since active surveillance for MDR-E was not consistent throughout the study period, all admitted newborns may not have been included in this study.

## Conclusion

This study showed a high prevalence of MDR-E intestinal carriage, multiple antibiotic resistance profiles, and a diversity of encoding resistance genes in our NICU. This situation required the development of antimicrobial stewardship initiatives as well as the maintaining of antimicrobial resistance surveillance systems. In addition, the knowledge of risk factor profiles can lead to the development of strategies to prevent colonization at all levels, the proper management of newborns colonized by MDRs can lead to the prevention of bloodstream infections and the occurrence of sepsis among these fragile patients.

## Supporting information

S1 Dataset (XLSX)
